# Unilateral External Fixator Combined with Lateral Auxiliary Frame for Ultimate Treatment of Tibia and Fibula Shaft Fractures with Poor Soft Tissue Conditions

**DOI:** 10.1155/2022/9990744

**Published:** 2022-08-05

**Authors:** Xinhui Wang, Bao Wang, Xizhi Hou, Xiaodong Cheng, Tao Zhang

**Affiliations:** ^1^Department of Orthopaedic Surgery, The Third Hospital of Hebei Medical University, Shijiazhuang, China; ^2^Department of Orthopaedic Surgery, The Third Hospital of Shijiazhuang City, Shijiazhuang, China; ^3^Key Laboratory of Biomechanics of Hebei Province, The Third Hospital of Hebei Medical University, Shijiazhuang, China

## Abstract

**Background:**

For severe soft tissue damage or open fracture, unilateral external fixation is one of the treatment choices. In the current study, a unilateral external fixator combined with a lateral auxiliary frame was used to treat tibia and fibula shaft fractures with poor soft tissue conditions to verify its feasibility for the ultimate treatment.

**Methods:**

We retrospectively analyzed the patients with tibia and fibula shaft fractures who underwent unilateral external fixator combined with lateral auxiliary frame between December 2018 and October 2020. The clinical outcomes were recorded.

**Results:**

31 patients with tibia and fibula shaft fractures who received unilateral external fixator combined with lateral auxiliary frame were included in the current study. Among them, 23 cases had closed fractures with poor soft tissue and 8 cases had Gastilo type I open fractures. The average duration of hospital stay was 7.3 ± 2.3 days. The causes of injury were traffic accidents in 15 cases (48.4%), fall from height in 7 cases (22.6%), crush injury in 5 cases (16.1%), and other causes in 4 cases (12.9%). During follow-up, the clinical healing time was 3.0 ± 0.85 months. Additionally, the infection rate of pin-tract and reoperation rate was 12.9% and 3.2%. Fortunately, all patients achieved fracture healing and recovered well without joint dysfunction and obvious claudication. The Johner-Wruh scores showed that 27 cases (87.1%) were “excellent” and 4 cases (12.9%) were “good.”

**Conclusions:**

The unilateral external fixator combined with lateral auxiliary frame is an effective option for ultimate treatment of the tibia and fibula shaft fractures with poor soft tissue conditions.

## 1. Introduction

Tibia and fibula fractures are the most common long bone fractures of the lower limb [1, 2]. Due to its special structure, fractures are often accompanied by severe soft tissue damage or formed into open fractures, especially tibia and fibula shaft fractures [3]. For poor soft tissue conditions or open tibia and fibula fractures, open reduction and internal fixation with bone plate often cause further damage to the soft tissues, thereby leading to catastrophic consequences such as soft tissue infection, necrosis, and even osteomyelitis [4]. The emergence of unreamed intramedullary nail technology can significantly improve the treatment effect of the tibia and fibula fractures with severe soft tissue damage, reduce surgery-related complications, and infection and expand internal fixation surgery indications, which attracts more and more attention [5–7]. However, unreamed intramedullary nail technology may lead to the decrease of the stability of the fracture end, and then, bone nonunion occurs [8]. Therefore, the reliable surgical treatment for the tibia and fibula shaft fractures with poor soft tissue conditions is urgently needed.

External fixators are deemed as osteosynthesis devices for management of severe soft tissue damage and open fractures with the advantages of less effect on the blood supply and invasion, and easy installation, flexible fixation [9, 10]. At first, external fixation was used as a temporary device and later developed as the ultimate treatment [11]. Apart from that, previous studies have attempted the external fixation for ultimate treatment of open fractures and it turns out that satisfactory outcomes are obtained [12, 13]. Correspondingly, Anjum et al. [14] have shown that unilateral external fixator for ultimate treatment of tibia and fibula shaft fractures can greatly shorten the operation time, reduce surgical trauma, and promote early recovery. However, external fixators have several complications in the clinical practice including pin-tract infection, nonunion, malunion, and refracture [15, 16]. With regard to these complications, it is widely believed to be associated with the mechanical properties of the fixators [17, 18], indicating that it is essential to explore an optimum prototype of external fixator for the tibia and fibula shaft fractures to reduce postoperative complications.

The current study is aimed at trying the unilateral external fixator combined with lateral auxiliary frame for ultimate treatment of the tibia and fibula shaft fractures with poor soft tissue conditions and then verifying the feasibility of this technique.

## 2. Materials and Methods

### 2.1. Patients

The study was retrospectively included the patients with tibia and fibula shaft fractures who underwent unilateral external fixator combined with lateral auxiliary frame between December 2018 and October 2020 at our hospital. Inclusion criteria were patients who (1) were aged from 18 to 65 years with tibia and fibula shaft fractures and (2) had poor soft tissue conditions, including closed fractures with extensive skin abrasions, skin necrosis, or localized multiple blisters or Gastilo type I open fractures. Exclusion criteria were patients who (1) had severe combined injuries or other lower limb fractures, (2) had Gustilo Type II/III open fracture with soft tissue defect, (3) had other serious medical diseases, and (4) refused external fixation treatment or were unable to cooperate with follow-up.

### 2.2. Surgery Procedure

All patients received general anesthesia and then were placed in supine position. After incision with a No. 11 or No. 15 blade, the drilled holes were made using 4.5 mm drill bit in the distal and proximal ends of the anterior medial tibia, and then, a 6 mm half-pin was screwed in each. The distal and proximal connecting caps were tightened after restoring the length and rotation of the lower limbs. Determining the fracture position under fluoroscopy, Kirschner wire was penetrated and reduction of the fracture was used by joystick technology. After reduction, a 6 -mm half-pin was inserted at the 2 cm distal and proximal end of the fracture to fix the fracture firmly. Afterwards, a half-pin was added to the distal and proximal bone masses to increase stability according to the situation, or not if the patient's bone quality was good. The external fixation rod was placed as close to the skin as possible to avoid soft tissue stimulation. When fracture reduction was satisfactory, a set of lateral auxiliary frame was added to the outside. The lateral auxiliary frame requires only two screws. Of these, one was penetrated through the Gerdy tubercle, and the other was screwed from lateral malleolus through inferior tibiofibular syndesmosis.

### 2.3. Postoperative Management

After surgery, antibiotics were intravenously injected for 48 hours. At day 2 postoperation, patients were guided to perform nonweight-bearing exercises on the premise that the pain was tolerable. At day 3 after operation, patients were instructed to walk on crutches. Additionally, patients needed to use the alcohol for care daily in order to avoid pin-tract infection. According to the reexamination 1-2 months after operation, patients were guided to walk with full weight-bearing gradually. When patients can walk with weight-bearing, auxiliary external fixator was removed. Then, according to fracture healing, half-pins were gradually removed in 2-3 times until they were completely removed.

### 2.4. Clinical Outcomes

The visual analogue scale (VAS) was used to evaluate the pain at preoperation and postoperative 3 days and 1 month. The lower extremity functional scale (LEFS) was unitized to assess the patient's recovery at 3, 6, and 12 months after surgery. The clinical healing time was defined as the dense callus formation at the fracture site, and the patient can walk with full weight-bearing without pain. At the last follow-up, the patient's recovery was evaluated according to the Johner-Wruh system [19].

### 2.5. Statistical Analysis

Data were analyzed using SPSS 19.0 software. The categorical variables were expressed as number (percentage), and the measurable variables were expressed as mean ± standard deviation (SD). The comparison of VAS and LEFS were conducted using one-way repeated measures ANOVA. When ANOVA showed a significant difference, post hoc analysis was conducted by LSD test. *P* < 0.05 was deemed as the significant difference.

## 3. Results

31 patients with tibia and fibula shaft fractures who received unilateral external fixator combined with lateral auxiliary frame were included in the current study. Patient characteristics were shown in Table 1. The average age was 36.5 ± 12.9 years and average duration of hospital stay was 7.3 ± 2.3 days. There were 22 males and 9 females. Of these, 17 of the tibia and fibula shaft fractures were on the left side and 14 cases on the right side. 23 cases had closed fractures and 8 cases had Gastilo type I open fractures. The causes of injury were traffic accidents in 15 cases (48.4%), fall from height in 7 cases (22.6%), crush injury in 5 cases (16.1%), and other causes in 4 cases (12.9%).

During follow-up, the clinical healing time was 3.0 ± 0.85 months. Additionally, we found that the infection rate of pin-tract was 12.9% (4 cases), and the reoperation rate was 3.2% (1 case). Briefly, 4 patients had external fixation pin tract redness, swelling, and exudation. Among which, a 33-year-old woman was injured in a traffic accident, and a 56-year-old woman suffered a crush injury. These two patients were treated with oral antibiotics combined with pin-tract care, and finally, the infection was controlled without affecting the recovery. One case was a 38-year-old male who was injured in a traffic accident and had pin-tract infection of the lateral auxiliary external fixator and improved after the removal. Another patient, a 63-year-old male, was injured in a traffic accident. He received a second operation to adjust the external fixator due to the loosening caused by pin-tract infection. The weight-bearing time was appropriately postponed, and the fracture finally healed. Fortunately, all patients achieved fracture healing and recovered well without joint dysfunction and obvious claudication. Representative images of good recovery after operation using unilateral external fixator combined with lateral auxiliary frame were shown in Figures 1 and 2. The Johner-Wruh scores showed that 27 cases (87.1%) were “excellent” and 4 cases (12.9%) were “good” (Table 1).

The average VAS scores were shown in Table 2, and the average VAS score at 3 days after operation was lower than the preoperative score (*P* < 0.001). At 1 month of postoperation, the VAS score was significantly decreased again (*P* < 0.001). As shown in Table 3, LEFS scores increased with the increase of post-operative time (*P* < 0.001).

## 4. Discussion

Previous studies have demonstrated that optimum configuration, fixation strength, and pin-tract infection are the main factors that hinder the wide acceptance of unilateral external fixation as ultimate treatment [20, 21]. Here, we introduced a method of unilateral external fixator combined with lateral auxiliary frame and tried to use it as the ultimate treatment for tibia and fibula shaft fractures with poor soft tissue conditions. Fortunately, all patients achieved benefit outcomes.

As we know, pin-tract infection cannot be effectively controlled, which will cause the external fixation needle to loosen and eventually lead to failure [22]. In the clinical application of unilateral external fixation, pin-tract infection rates reported by previous studies vary. For instance, Parameswaran et al. [23] have analyzed the outcomes using external fixation and found that pin-tract infection rate is almost 11.2%. Another study has reported that the pin-tract infection rate is even as high as 52% in pediatric patients underwent external fixation [24]. For pin-tract infection, serval scholars have considered that stability, material, and the type of the external fixator, the technique of pin placement, and the care of the pin-tract are closely associated with pin-tract infection [17, 21, 25]. In our study, pin-tract infection was in 4 cases; however, it was improved after oral antibiotics or adjustment of external fixator. The satisfactory outcomes in the current study may be closely related to strict adherence to half-pin placement technology. The previous study has demonstrated that correct technique is helpful to prevent the pin-tract infection including drill placement and declination of local temperature during predrilling process [26]. Additionally, half-pins were screwed in the weaker soft tissues to reduce irritation to muscles and tendons, which consistent with a previous study that repeated stimulation of the muscles leads to local microbleeding and inflammation, thereby causing pin-tract infections [20]. Moreover, in the current study, the screws of the unilateral external fixator were penetrated from the anterior and medial surface of the tibia, while the two screws of the lateral auxiliary frame were, respectively, penetrated from the Gerdy tubercle and the lateral malleolus. This improved nail placement technique can reduce the irritation to soft tissues, and it may be one of the main reasons for the effective reduction of pin-tract infection in this study. Those findings suggested that using the correct technique combined with postoperative care in the unilateral external fixation process exert the key roles on good recovery.

A reasonable unilateral external fixation configuration can provide proper stability for the entire process of fracture healing, which is the key to the ultimate success of treatment [27, 28]. In this study, we adopted a new method (unilateral external fixator combined with lateral auxiliary frame) for treating the tibia and fibula shaft fractures in order to obtain better fixation strength and provide a prerequisite for fracture healing. Delayed union or nonunion may occur if the strength of the external fixator is insufficient. A study by Wu et al. [29] has shown that there may be high bending stress at the nail-bone contact, especially for unilateral fixators. High stress can cause bone resorption or necrosis and may lead to pin loosening, which can affect the fixation strength, thereby affecting bone healing. And pure unilateral external fixators provide lower fixation strength, which may lead to increased pinning problems, which further lead to delayed healing. In addition, higher-strength external fixation does not cause postunion osteopenia as plate fixation. The research results of Chao et al. [30] also suggested that adjusting the strength of the external fixator can promote fracture healing.

In the preliminary study, we designed 9 common configurations for the tibia and fibular shaft fractures. The schematic diagram of 9 configurations of unilateral external fixation guided by finite element analysis for the tibia and fibula shaft fractures were shown in Figure 3. Of these, 9 kinds of configurations included 7 configurations of single unilateral external fixator, and h and i configurations with additional lateral auxiliary frame. Maximum displacements of 9 configurations under vertical load were shown in Figure 4. After adding a vertical load of 600 N, the maximum displacement was recorded. After analyzing the displacement data, we found that spreading the screws, increasing the number of screws, and shortening the distance between the bone and the external fixator rod can effectively increase the fixation strength of the unilateral external fixation. In addition, adding an auxiliary frame on the outside can significantly increase the fixing strength, especially the lateral auxiliary frame. Consistently, Skomoroshko et al. [31] have revealed that displacement of 0.2-1 mm is considered to be beneficial; however, more than 2.0 mm can lead to poor outcomes. In the clinical application of unilateral external fixator combined with a lateral auxiliary frame, we found that the clinical healing time was 3.0 ± 0.85 months, and no patient had loosening of external fixation due to weight-bearing. Importantly, the main reason of using clinical healing time instead of fracture healing time in the current study was to avoid the refracture risk caused by premature removal of the external fixator. In our best knowledge, external fixation has a higher incidence of refracture in the treatment of the tibia and fibula shaft fractures, which is another major factor affecting the efficacy of external fixation [32, 33]. Greene et al. [34] have pointed out that local pressure stimulation can effectively promote bone formation and calcium accumulation. Thus, gradually increasing weight-bearing under the protection of external fixation may be an effective means to avoid refracture. In our study, half-pins were gradually removed in 2-3 times, and weight-bearing was gradually increased. Fortunately, none of patients had refracture, indicating that half-pin removal gradually can effectively avoid the occurrence of refracture.

In this study, the patient's VAS score of 3.8 ± 1.2 at 3 days after surgery was significantly lower than the preoperative score of 7.1 ± 1.3, and the VAS score dropped to 1.0 ± 1.2 one month after surgery. This result proved that the unilateral external fixator combined with the lateral auxiliary frame can effectively and quickly relieve the pain of the affected limb. Due to the rapid relief of postoperative pain, patients can perform knee and ankle functional exercises on the second day after surgery, thereby avoiding traumatic foot drop and joint stiffness. LEFS is considered as the reliable indicator to assess functional mobility [35]. Our study showed that LEFS was significantly increased at postoperative 6 months compared with 3 months after operation, indicating that the clinical healing time was 3-6 months. At postoperative 12 months, the LEFS score of 75.2 ± 3.7 was satisfactory. Additionally, The Johner-Wruh score was excellent in 87.1% and good in 12.9% one year after the operation, which proved that its clinical efficiency was also satisfactory, supplementing the short board of the LEFS score in clinical efficacy evaluation.

The limitation of this study lies in the single-arm study with a single center and small sample. Gustilo Type II/III was excluded to avoid the soft tissue factors in the study. In the future, we will increase sample size to verify the efficacy of the new unilateral external fixation configuration and attempt the treatment for the Gustilo Type II/III open tibia and fibula shaft fractures. This study focused more on the difference in fixation strength caused by the external fixation configuration, but there is no direct data to prove the effect of different fixation strength on fracture healing. In future studies, our team will design animal experiments to demonstrate the positive effect of changing the fixation strength of unilateral external fixation on fracture healing.

## 5. Conclusion

A unilateral external fixator combined with lateral auxiliary frame can accelerate bone healing, shorten the treatment time, allow early functional exercise, and reduce complications; therefore, it is an option for ultimate treatment of the tibia and fibula shaft fractures with poor soft tissue conditions.

## Figures and Tables

**Figure 1:** Representative images of good recovery after operation using unilateral external fixator combined with lateral auxiliary frame. The X-ray images at preoperation (a, b), after operation (c, d), postoperative 3 months (e, f), postoperative 6 months (g, h), and 12 months (i, j), respectively.

**Figure 2:** Representative images of good recovery after operation using unilateral external fixator combined with lateral auxiliary frame. The X-ray images at preoperation (a, b), after operation (c, d), postoperative 3 months (e, f), postoperative 6 months (g, h), and12 months (i, j), respectively.

**Figure 3:** Schematic diagram of 9 configurations of unilateral external fixation guided by finite element analysis for tibia and fibula shaft fractures. (a) Classical configuration, all external fixation pins were located in the same plane, following the principle of “near-near, far-far” in the fracture site. (b) Reducing the distance between connecting rod to shafts. (c) Increasing distance between connecting rod to shafts. (d) Half-pins were placed away from the fracture end. (e) Half-pins were placed close to the fracture end. (f) Increase the number of half-pins on a single fracture segment. (g) Several half-pins are inserted at different angles. (h) A set of additional lateral auxiliary frame were inserted into the anterior tibia crest from anterior tibia. (i) A set of additional lateral auxiliary frame were penetrated through the Gerdy tubercle and the lateral malleolus.

**Figure 4:** Maximum displacements of 9 configurations under vertical load. (a) 2.199 mm. (b) 2.165 mm. (c) 5.672 mm. (d) 4.963 mm. (e) 2.294 mm. (f) 2.063 mm. (g) 2.048 mm. (h) 1.508 mm. (i) 0.673 mm.

**Table 1:** Patient characteristics.

Case	Age (years)	Gender	Fracture side	Injury causes	Duration of hospital (days)	Reoperation	Clinical healing time (months)	Complications	Johner-Wruh score
1	24	Male	Left	Traffic accident	5	No	2	No	Excellent
2	33	Female	Right	Traffic accident	7	No	3	Pin-tract infection (oral antibiotics)	Excellent
3	25	Male	Left	Traffic accident	11	No	2	No	Excellent
4	36	Male	Left	Fall from height	6	No	3	No	Excellent
5	43	Female	Right	Traffic accident	5	No	4	No	Good
6	55	Female	Left	Fall from height	5	No	3	No	Good
7	61	Male	Right	Traffic accident	4	No	5	No	Excellent
8	19	Female	Left	Crush injury	7	No	2	No	Excellent
9	63	Male	Left	Traffic accident	11	Yes	5	Pin-tract infection (adjust the external fixator)	Good
10	37	Male	Right	Fall from height	8	No	3	No	Excellent
11	28	Male	Right	Crush injury	5	No	2.5	No	Excellent
12	29	Male	Left	Crush injury	9	No	4	No	Excellent
13	43	Male	Left	Traffic accident	10	No	3	No	Excellent
14	58	Male	Right	Other	4	No	4	No	Excellent
15	21	Male	Left	Crush injury	8	No	2	No	Excellent
16	47	Male	Right	Other	7	No	3	No	Good
17	35	Male	Left	Fall from height	12	No	3	No	Excellent
18	31	Female	Right	Other	10	No	3	No	Excellent
19	28	Male	Left	Traffic accident	8	No	2.5	No	Excellent
20	56	Female	Right	Crush injury	5	No	4	Pin-tract infection (oral antibiotics)	Excellent
21	36	Male	Left	Traffic accident	5	No	3	No	Excellent
22	44	Male	Right	Traffic accident	11	No	4	No	Excellent
23	27	Male	Left	Other	6	No	2.5	No	Excellent
24	32	Female	Right	Fall from height	7	No	2.5	No	Excellent
25	55	Male	Left	Traffic accident	9	No	3	No	Excellent
26	26	Female	Right	Fall from height	6	No	2.5	No	Excellent
27	38	Male	Right	Traffic accident	10	No	4	Pin-tract infection (removal auxiliary external fixator)	Excellent
28	20	Male	Left	Traffic accident	5	No	2	No	Excellent
29	33	Female	Right	Fall from height	6	No	2.5	No	Excellent
30	23	Male	Left	Traffic accident	8	No	2.5	No	Excellent
31	24	Male	Left	Traffic accident	5	No	2	No	Excellent

**Table 2:** Comparison of VAS score between preoperation and postoperation.

Preoperation	Postoperative 3 days	Postoperative 1 month	*F* value	*P* value
7.1 ± 1.3	3.8 ± 1.2^∗∗^	1.0 ± 1.2^∗∗^^##^	181.4	<0.001

There were differences in VAS scores between different measurement time points. ^∗∗^*P* < 0.01 vs. preoperation; ^##^*P* < 0.01 vs. postoperative 3 days. VAS: visual analogue scale.

**Table 3:** Comparison of LEFS score between postoperative 3 months and postoperation 12 month.

Postoperative 3 months	Postoperative 6 months	Postoperative 12 months	*F* value	*P* value
35.5 ± 9.7	59.5 ± 4.2^∗∗^	75.2 ± 3.7^∗∗^^##^	296.0	<0.001

There are differences in LEFS at different measurement time points. ^∗∗^*P* < 0.01 vs. postoperative 3 months; ^##^*P* < 0.01 vs. postoperative 6 months. LEFS: lower extremity functional scale.

## Data Availability

All data generated or analyzed during this study are included in this article.

## Abbreviations

VAS: Visual analogue scale
LEFS: Lower extremity functional scale
SD: Standard deviation.
